# Metformin Ameliorates Senescence of Adipose-Derived Mesenchymal Stem Cells and Attenuates Osteoarthritis Progression via the AMPK-Dependent Autophagy Pathway

**DOI:** 10.1155/2022/4620254

**Published:** 2022-06-03

**Authors:** Zheng Li, Lin Liu, Yanni Yang, Haishi Zheng, Yongsong Cai, Yao Ma, Ruiying Gu, Ke Xu, Rui Zhang, Peng Xu

**Affiliations:** ^1^Department of Orthopedics, The First Affiliated Hospital of Xi'an Jiaotong University, Xi'an, China; ^2^Department of Joint Surgery, Honghui Hospital, Xi'an Jiaotong University, Xi'an, China; ^3^Department of Clinical Medicine of Traditional Chinese and Western Medicine, Shaanxi University of Chinese Medicine, Xianyang, China; ^4^Department of Biochemistry and Molecular Biology, School of Basic Medical Science, Xi'an Jiaotong University, Xi'an, China; ^5^Translational Medicine Center, Honghui Hospital, Xi'an Jiaotong University, Xi'an, China

## Abstract

Osteoarthritis (OA) is one of the most serious age-related diseases worldwide that drastically affects the quality of life of patients. Despite advancements in the treatment of arthritis, especially with adipose-derived mesenchymal stem cells (ADSCs), senescence-induced alterations in ADSCs negatively affect the treatment outcomes. This study was aimed at mechanistically exploring whether metformin could ameliorate the senescence of ADSCs and at exploring the effect of metformin-preconditioned ADSCs in an experimental OA mouse model. In this study, an H_2_O_2_-induced mouse ADSC senescent model was established. Cell proliferation, senescence, and autophagy were investigated in vitro. Moreover, the effects of intra-articular injection of metformin-preconditioned ADSCs were investigated in vivo. Metformin could promote autophagy and activate the AMPK/mTOR pathway in ADSCs. The metformin-enhanced autophagy could improve the survival and reduce the senescence of ADSCs. The protective effects of metformin against senescence were partially blocked by 3-methyladenine and compound C. Injection of metformin-preconditioned ADSCs slowed OA progression and reduced OA pain in mice. The results suggest that metformin activates the AMPK/mTOR-dependent autophagy pathway in ADSCs against H_2_O_2_-induced senescence, while metformin-preconditioned ADSCs can potentially inhibit OA progression.

## 1. Introduction

Osteoarthritis (OA) is a prevalent degenerative joint disease, with aging, trauma, and obesity identified as significant risk factors [1]. In addition to affecting the elderly, it also affects other populations [2]. Apart from persistent pain and disability to patients, OA results in substantial global health and economic burden to society.

OA is characterized by irreversible articular cartilage degeneration, synovial inflammation, and subchondral bone remodeling [3, 4]. Currently available strategies can neither delay nor prevent the pathophysiology of OA, and symptomatic improvement and eventual total knee arthroplasty surgery are the standards of care. Despite advancements in OA treatment, effective and reasonable disease-modifying therapies are lacking.

Mesenchymal stem cell (MSC) therapy represents a promising treatment modality for experimental and clinical OA therapeutic applications [5, 6] . Adipose-derived mesenchymal stem cells (ADSCs) can be easily isolated, and they exhibit anti-inflammatory, immunomodulatory, and chondrometabolic regulation effects in joint tissues [7]; therefore, they may be used in OA treatment.

However, despite their great therapeutic value, when ADSCs are subjected to oxidative stress or multiple expansion, they undergo cellular senescence with reduction of therapeutic efficacy and survival rate, as shown by decreased proliferation, impaired cellular differentiation, and increased senescence-associated secretory phenotype [8]. Cellular senescence is identified as an inescapable and irreversible state that occurs when cells are exposed to numerous stress stimuli [9]. Stem cell aging not only results in the degeneration of the body or organs; moreover, the function of stem cells also changes with aging, reducing their potential in treating diseases. While healthy and dynamic stem cells play a promising role, senescence-induced alterations are thought to be the major hurdle in the clinical application of ADSC therapy [8]. Therefore, exploring an effective strategy to prevent ADSC senescence is meaningful for applying ADSC therapy for OA.

Although the application of stem cells for promoting tissue regeneration and repair has been extensively studied, and the topic of stem cell aging has become popular in recent years, little is known about the aging regulation mechanism. Autophagy plays a cytoprotective role in the degradation of malfunctioning organelles and proteins under different conditions [10]. Senescence and autophagy are essential for bioenergetic homeostasis [11]. Enhanced autophagy protects stem cells from senescence, while reduced autophagy causes cell senescence [12]. Autophagy intervention is a potential therapeutic target to rejuvenate stem cells [8].

Many proteins are involved in autophagy. Mammalian target of rapamycin (mTOR) is involved in maintaining cellular homeostasis, which is closely related to autophagy [13]. Adenosine monophosphate-activated protein kinase (AMPK) is a key molecule required for autophagy regulation, whose downstream protein is mTOR [14]. Thus, regulation of autophagy through the AMPK/mTOR pathway becomes a reasonable target for the prevention of stem cell senescence.

Metformin is a first-line treatment agent for diabetes. It is known to influence not only cellular metabolic processes but also inflammation, oxidative damage, diminished autophagy, cell senescence, and apoptosis [15, 16]. The beneficial role of metformin in targeting multiple mechanisms of aging has been extensively studied. Metformin regulates cell homeostasis primarily through the AMPK-dependent signaling pathways [15]. Herein, we evaluated the effects of metformin on H_2_O_2_-induced senescence of ADSCs and investigated the underlying mechanism, especially, the AMPK/mTOR-dependent autophagy pathway. We also demonstrated the beneficial effects of injecting metformin-preconditioned ADSCs in an experimental OA mouse model.

## 2. Materials and Methods

### 2.1. Preparation and Characterization of ADSCs

ADSCs derived from murine inguinal adipose tissue were collected and characterized. Briefly, fat tissue was isolated aseptically from healthy C57BL/6 mice (6–8 weeks; male) after anesthesia, washed with phosphate-buffered saline (PBS), minced, and mixed with collagenase type I (Sigma-Aldrich, St. Louis, MO, USA). Next, the mixture was intermittently shaken for 50 min at 37°C. After centrifugation at 1000 rpm for 5 min, the supernatant and adipose suspension were discarded. ADSCs were suspended in complete medium containing F12/DMEM (HyClone, Logan, UT, USA), containing 10% fetal bovine serum (Gibco, Melbourne, Australia) and 1% penicillin/streptomycin (HyClone). The cells of passages 3–6 were utilized for subsequent experiments.

The immunophenotypes of ADSCs were determined by flow cytometry. The cells were incubated with the following primary antibodies for 30 min: CD105 (Abcam, Cambridge, UK), CD34 (Thermo Fisher Scientific, Massachusetts, USA), CD29, CD90, and CD45 (BioLegend, San Diego, USA). The corresponding isotype antibodies replaced the primary antibodies as negative control. After washing twice, the cells were resuspended for flow cytometric analysis (Beckman, USA). Data were analyzed using the EXPO32-ADC software.

The trilineage differentiation of ADSCs was evaluated by culturing them in adipogenic, osteogenic, and chondrogenic induction media (Haixing Biosciences, Suzhou, China). After 2–3 weeks, the cells were separately stained with alizarin red, oil red O, and toluidine blue solutions.

### 2.2. Cell Proliferation Assay

Cell viabilities were assessed using a Cell Counting Kit-8 (CCK-8) (Beyotime, China). Following the manufacturer's protocol, ADSCs were seeded in 96-well culture plates with 3000 cells per well. Subsequently, the cells were treated with various concentrations of specified drugs for an appropriate time. A total of 10 *μ*L of the CCK-8 reagent was added to each well and incubated at 37°C for 1 h. Lastly, the absorbance was measured at 450 nm using a microplate spectrophotometer (Thermo Fisher Scientific).

### 2.3. Treatments with H_2_O_2_, Metformin, and Antagonists

Cellular senescence was induced by exposing about half the density of ADSCs to H_2_O_2_ for 2 h. After removal of H_2_O_2_, the cells were recultured in fresh growth medium. The effectiveness of metformin pretreatment on preventing cellular senescence was studied by incubating the cells with specific antagonists of autophagy and AMPK: 3-methyladenine (3-MA; 5 mM; Sigma-Aldrich) and compound C (10 *μ*M; MedChemExpress, Shanghai, China) diluted in growth medium. ADSCs were pretreated with 100 *μ*M metformin (Sigma-Aldrich) for 24 h, followed by exposure to 200 *μ*M H_2_O_2_ for 2 h. The cells were then recultured in fresh growth medium.

### 2.4. SA-*β*-Gal Staining

ADSC senescence was investigated by staining them with SA-*β*-Gal (Beyotime) according to the manufacturer's protocol. The cells were incubated in a fixation buffer for 15 min at room temperature. After washing twice with PBS, the samples were incubated with SA-*β*-Gal staining solution without CO_2_ for at least 12 h at 37°C. SA-*β*-Gal-positive cells stained in blue were randomly captured using an inverted microscope (Leica, Germany). Further quantification and statistical analysis were performed.

### 2.5. Transmission Electron Microscopy

Transmission electron microscopy was performed to verify autophagosome formation. The cells were fixed with 3% glutaraldehyde solution overnight. After fixation, the samples were postfixed in 2% osmic acid for 1 h, stained with 2% uranyl acetate for 1 h, and dehydrated with increasing concentrations of ethanol. The samples were embedded in Araldite and stained with lead citrate and then cut into ultrathin sections. Finally, the sections were photographed under a transmission electron microscope (H-7650, Hitachi, Tokyo, Japan).

### 2.6. ROS Detection

The cellular ROS levels were measured using an ROS assay kit (Beyotime). Briefly, the cells were washed with PBS after treatment as previously described and then incubated with 10 *μ*mol DCFH-DA for 20 min at 37°C. Afterward, the cells were washed thrice with serum-free medium, and the fluorescence was analyzed by a fluorescence microscope (Leica, Germany). Moreover, the cells were analyzed by flow cytometry (Beckman, USA). The mean fluorescence intensity (MFI) of DCF represented the ROS level.

### 2.7. Immunofluorescence Staining

Briefly, the cells on slides were immobilized using 4% paraformaldehyde and permeabilized using 0.1% Triton X-100 in PBS. Then, the cells were blocked using goat serum (Zhongshan Golden Bridge, China) and incubated overnight at 4°C with anti-*γ*H2A.X antibody (Cell Signaling, MA, USA, 1 : 500). After washing, the cells were incubated with goat anti-rabbit Alexa Fluor 594 (Abcam, UK, 1 : 1000). The cells were then counterstained with 4′,6-diamidino-2-phenylindole (DAPI, Bioworld, China, 1 : 2000) for 5 min. The slides were imaged using a fluorescence microscope (Leica, Germany).

### 2.8. Western Blotting

Cellular protein was extracted using RIPA buffer (Beyotime) containing phenylmethylsulfonyl fluoride and phosphatase inhibitors. Equal amounts of extracted cellular protein were resolved on 6–12% SDS-PAGE-denaturing gels and transferred electrophoretically onto polyvinylidene difluoride membranes. The membranes were blocked with 5% no-fat milk for 2 h at room temperature. The bands were incubated with the following diluted primary antibodies: p-AMPK, AMPK, p-mTOR, mTOR, Beclin-1, LC3B, *γ*H2A.X (Cell Signaling, MA, USA, 1 : 1000), P21, P16 (Abcam, Cambridge, UK, 1 : 1000), Rad51 (Abcam, UK, 1 : 5000), and *β*-actin (Boster, Wuhan, China, 1 : 5000) overnight at 4°C. After washing three times with TBST, the membranes were then incubated for 2 h at room temperature with goat anti-rabbit or anti-mouse secondary antibodies (Boster, Wuhan, China, 1 : 5000). The excessive secondary antibody was washed off three times with TBST, and the bands were visualized using the Bio-Rad imaging system with the ECL imaging kit (Millipore Corporation). The intensity of the images was quantified by using ImageJ software.

### 2.9. OA Induction and Treatment

C57BL/6 mice were purchased from Xi'an Jiaotong University and utilized for all experiments. The mice were maintained in an accredited facility and received a standard diet and tap water. The experiments were approved by the Institutional Animal Care and Use Committee of Xi'an Jiaotong University.

The 12-week-old male C57BL/6 mice were randomly assigned to four groups (12 mice each): OA, OA+ADSCs, OA+metformin-preconditioned ADSCs, and sham. Male mice are more suitable than female mice for evaluating the experimental effects following destabilization of the medial meniscus (DMM) [17, 18]. Mice in all groups except for the sham group were subjected to DMM in the right knee joints. The mice were first anesthetized with inhalational isoflurane and intraperitoneal injection of sodium pentobarbital (10 mg/mL and 0.5 mL/100 g). After anesthesia, medial parapatellar arthrotomy was performed. After dissection of the anterior fat pad, the medial meniscotibial ligament was identified and transected. The patella was reset, and the incisions of the capsule and skin were neatly closed with sutures. The sham group was subjected to only a medial capsulotomy. Intra-articular cell transplantation was randomly allocated to mice receiving DMM surgery. Metformin-preconditioned or not preconditioned ADSCs (2 × 10^4^) were injected (10 *μ*L per joint) using a microliter syringe and 26s-gauge needles (Hamilton Company) every two weeks starting from four weeks after DMM surgery. After 12 weeks of OA induction, the mice were euthanized, and the right knee joints were isolated.

### 2.10. ADSC Labelling and In Vivo Imaging Tracking

ADSCs were labelled in vitro with DiR (DiIC18(7)1,1'-dioctadecyltetramethyl indotricarbocyanine iodide) (Beijing Fluorescence, China). Briefly, the cell density was adjusted to 1 × 10^6^, and then, the cells were incubated with 62.5 *μ*g/mL DiR at 37°C for 30 min. After this, the cells were centrifuged and washed with PBS. The fate of the injected ADSCs was monitored at 1, 3, and 7 days using a small animal in vivo imaging system (Vieworks, Korea). The fluorescence region represented the region of interest.

### 2.11. Microcomputed Tomography (CT) Analysis

The right knee joints were analyzed by micro-CT (Y Cheetah, Germany). The scanning was conducted using a voltage of 80 kV and a current of 35 *μ*A with a resolution of 6 *μ*m. The scans were reconstructed and analyzed in VGStudio MAX 2.4.0 software (Volume Graphics, Heidelberg, Germany). The region of interest was modulated in the tibial subchondral bone. Average bone volume fraction (BV/TV), trabecular thickness (Tb.Th), trabecular number (Tb.N), and trabecular separation (Tb.Sp) were analyzed using standardized parameters.

### 2.12. Histology and Immunohistochemistry Analysis

The right knee joints of mice were fixed in 4% buffered paraformaldehyde for two days. Then, the samples were decalcified in 10% ethylenediaminetetraacetic acid solution for three weeks. The paraffin blocks were coronally cut into sections with 6 *μ*m thickness. The sections were deparaffinized, dehydrated, and processed for hematoxylin and eosin (H&E) and Safranin O and Fast Green staining. Immunohistochemistry was performed according to a standard protocol. The sections were separately incubated with mouse anti-COL2A1 (Santa Cruz Biotechnology, Texas, USA, 1 : 50), rabbit anti-MMP-13 (Bioss, Beijing, China, 1 : 200), rabbit anti-F4/80 (Cell Signaling, 1: 400), rabbit anti-iNOS (Abcam, 1 : 100), and rabbit anti-CD206 (Abcam, 1 : 1000) overnight at 4°C. Then, the slides were incubated with a biotin-labeled IgG secondary antibody (Zhongshan Golden Bridge, Beijing, China) and stained with a diaminobenzidine (DAB) substrate and counterstained with hematoxylin. Cartilage degradation and synovitis were evaluated using the Osteoarthritis Research Society International (OARSI) scoring system by two independent observers blinded to treatment [19].

### 2.13. Pain Behavioral Measurement

Catwalk-automated gait analysis was used to assess the OA-associated pain by using the Catwalk XT 9.0 system (Noldus Information Technology, Wageningen, Netherlands). The testing was performed before and 12 weeks after the DMM operation by two independent experimenters blinded to treatment. The mice were acclimated to the walkway one day before the day of assessment. Each freely moving mouse was placed individually on a platform. The mice were allowed to walk voluntarily back and forth. The paw prints were automatically captured with a video camera.

Paw print area, max contact area, max contact max intensity, duty cycle, mean intensity, stand, and swing speed were analyzed. The ratio of right hind to left hind of the parameters was calculated as previously described [20].

### 2.14. Statistical Analysis

All experiments in vitro were independently representative at least triplicates. The data are expressed as the mean ± standard deviation (SD). Statistical analysis was conducted using GraphPad Prism version 8.0 (GraphPad Software, San Diego, CA, USA). ANOVA following by Tukey's test was appropriately used to compare multiple groups. Statistical difference was considered significant when the *p* value was less than 0.05.

## 3. Results

### 3.1. Metformin Protected ADSCs from H_2_O_2_-Induced Cell Senescence

We isolated ADSCs from the C57BL/6 inguinal fat pad adipose tissues. Their morphology (Figure 1(a)), osteogenic, adipogenic, and chondrogenic differentiation capacities are shown in Figure 1(b). Flow cytometric analysis for detecting ADSC markers revealed that the cells were positive for CD29, CD90, and CD105, but the expression of CD34 and CD45 was extremely low (Figure 1(c)).

To evaluate the influence of metformin on cell proliferation during long-term in vitro expansion, the proliferation capacity of ADSCs was assessed using the CCK-8 kit during in vitro culture. Metformin displayed no cytotoxic effects in ADSCs after 24 h treatment at concentrations of ≤5 mM (Figure 2(a)).

H_2_O_2_ was used to induce ADSC senescence according to a previous study. H_2_O_2_ significantly inhibited ADSC proliferation in a concentration-dependent manner starting at 200 *μ*M for 2 h (Figure 3(a)); therefore, the same concentration and time were chosen for subsequent experiments. Next, ADSCs were pretreated with metformin (50–400 *μ*M) for 24 h and then exposed to 200 *μ*M H_2_O_2_ for 2 h. Metformin at concentrations of 100 *μ*M and 200 *μ*M metformin was adequate to significantly protect ADSCs from the H_2_O_2_-induced cell viability loss (Figure 3(b)).

SA-*β*-Gal staining revealed that few senescent ADSCs were observed in the control group, while typical senescence was noted in the H_2_O_2_ group. However, the percentage of SA-*β*-Gal-positive cells in the metformin pretreatment group was significantly lower than that in the H_2_O_2_ group (Figure 3(c)).

Furthermore, p21 and p16 expression levels in the metformin-pretreated groups were lower than those in the H_2_O_2_ group (Figure 3(d)). The results showed that pretreatment with metformin could inhibit the aging of ADSCs.

### 3.2. Metformin Reversed the Excess ROS Production and DNA Damage Induced by H_2_O_2_

Cellular ROS levels were further analyzed as ROS plays a vital role in stem cell aging. The results showed a remarkably increased level of ROS after treatment with H_2_O_2_; the level of ROS was significantly reduced after pretreatment with metformin (Figures 4(a) and 4(b)). These findings revealed that pretreatment with metformin could inhibit ROS generation, which was induced by H_2_O_2_.

Considering DNA damage as a major feature of senescence, the well-known indicators, *γ*H2A.X and Rad51, were further quantified. Fluorescence imaging revealed the accumulation of *γ*H2A.X in ADSCs after H_2_O_2_ treatment, whereas the fluorescence intensity was decreased after metformin pretreatment (Figure 4(c)). As shown in Figure 4(d), corresponding with the result of immunofluorescence, western blot analysis indicated that the expression level of *γ*H2A.X was significantly increased after treatment with H_2_O_2_. Meanwhile, Rad51 was downregulated by H_2_O_2_. Taken together, these data suggested that metformin could also alleviate H_2_O_2_-induced cellular senescence, possibly by relieving ROS generation and DNA damage.

### 3.3. Autophagy Inhibition Blocked the Protective Effect of Metformin

Autophagy in H_2_O_2_-induced senescence was determined by monitoring autophagosome formation in each group using transmission electron microscopy. Autophagosomes were decreased in the cytoplasm of H_2_O_2_-induced senescent ADSCs. Metformin pretreatment significantly increased the number of autophagic vacuoles compared with the H_2_O_2_ group; however, when cotreated with 3-MA, the number of autophagic vacuoles decreased despite metformin pretreatment (Figure 5(a)).

The effect of metformin on autophagy was further verified by evaluating the expression levels of LC3B-II/LC3B-I and Beclin-1 through western blotting. As shown in Figure 5(b), metformin pretreatment increased the expression level of LC3B-II/LC3B-I and Beclin-1.

Whether metformin protected against H_2_O_2_-induced senescence by regulating autophagy was determined by cotreating ADSCs with metformin and 3-MA. Similar to the results of transmission electron microscopy, LC3B-II/LC3B-I and Beclin-1 levels decreased upon H_2_O_2_ exposure. In addition, LC3B-II/LC3B-I and Beclin-1 levels were significantly increased in the metformin pretreatment group, indicating that metformin promotes autophagy. However, LC3B-II/LC3B-I and Beclin-1 levels were lower in the group with metformin and 3-MA cotreatment than in the metformin pretreatment group (Figure 5(c)). These results indicated that metformin activated autophagy and then suppressed H_2_O_2_-induced senescence.

### 3.4. Role of AMPK/mTOR Signaling Pathway in Protecting ADSCs from Senescence

We investigated the signaling pathway that leads to the activation of autophagy by metformin. Metformin increased the level of AMPK phosphorylation and suppressed the level of mTOR phosphorylation in a concentration-dependent manner, starting at 50 *μ*M (Figure 6(a)). This indicated that metformin stimulated the AMPK/mTOR signaling pathway in ADSCs. Compared with normal ADSCs, the level of AMPK phosphorylation was downregulated and that of mTOR phosphorylation was upregulated in senescent ADSCs, suggesting that senescence in ADSCs proceeds through the AMPK/mTOR signaling pathway.

The regulatory effect of metformin on the AMPK-mediated autophagy signaling pathway was confirmed by pretreating ADSCs with the specific AMPK inhibitor compound C. Compound C increased the levels of p21, p16, and p-mTOR but decreased Beclin-1 levels and altered LC3B-II/LC3B-I and p-AMPK levels (Figure 6(b)). Thus, our results indicate that metformin conferred protection against H_2_O_2_-induced senescence by repressing the mTOR signaling pathway in an AMPK-mediated manner.

### 3.5. DiR-Labeled ADSCs Were Visualized in DMM-Induced Murine OA Model

The fate of the injected cells plays an important role in the treatment process. DiR-labeled ADSCs were observed using an *in vivo* imaging system. The knee joints of the mice showed significant fluorescence signal after injection. Although the fluorescence signals were reduced at 7 days postinjection, some fluorescence indicated that the stem cells were alive during this period (Figures 7(a) and 7(b)).

### 3.6. Metformin-Preconditioned ADSCs Showed Protective Effects in OA

#### 3.6.1. Articular Cartilage

The OA severity was scored according to the OARSI evaluation criteria, including maximal and summed scores. At 12 weeks postsurgery, the cartilage in the OA group exhibited severe degeneration (Figure 8(a)). The cartilage in ADSC and metformin-preconditioned ADSC groups exhibited moderate cartilage degeneration with a significantly lower OARSI score than that in the OA group (*p* < 0.05) (Figure 8(b)). Furthermore, the metformin-preconditioned ADSC group had a significantly lower summed score than the ADSC group (Figure 8(c)).

The effect of ADSCs on cartilage degradation was further verified by analyzing the expression of collagen II by immunohistochemical staining. The ADSC and metformin-preconditioned ADSC groups exhibited notably higher staining of collagen II than the OA group (Figure 9(a)). Although the level was apparently high in the metformin-preconditioned ADSC group and the ADSC group, the difference was not significant.

As natural collagenases, MMP-13, play pivotal roles in accelerating cartilage matrix degradation. The ADSC and metformin-preconditioned ADSC groups had lower percentages of chondrocytes positive for MMP-13 than the OA group (Figure 9(b)). These findings indicated that treatment with ADSCs (especially preconditioned with metformin) effectively protected the cartilage matrix against severe degradation.

#### 3.6.2. Synovium

Since it has been reported that synovial inflammation is strongly related to OA progression, synovial inflammatory responses were examined using H&E and immunohistochemical staining. In the OA model, synovium hyperplasia and infiltration of inflammatory cells were observed. However, treatment with ADSCs (preconditioned with metformin or not) showed a reduced degree of synovial inflammation and essentially prevented fibrotic deposition (Figure 10(a)).

Synovial inflammation is regulated by immune cells such as macrophages, neutrophils, and T cells [21]. Macrophages play a significant role in OA progression. The dysregulated balance between M1 and M2 macrophages is closely associated with OA severity. Immunohistochemistry staining showed that the levels of specific markers for macrophages (F4/80), M1 phenotype (iNOS), and M2 phenotype (CD206) were significantly increased in the synovial tissue at 12 weeks post-DMM surgery (Figures 10(b)–10(d)). However, F4/80 and iNOS levels significantly decreased and CD206 levels significantly increased in the groups treated with ADSCs and metformin-preconditioned ADSCs (Figures 10(b)–10(d)). Moreover, metformin significantly inhibited iNOS expression (Figure 10(c)).

Collectively, these results indicated that ADSCs effectively facilitate macrophage polarization to a homeostatic phenotype and that metformin-preconditioned ADSCs produce a better therapeutic effect than ADSCs in DMM-induced OA.

#### 3.6.3. Subchondral Bone

Pathological alterations in the subchondral bone also contribute to OA development [22]. Remarkable differences in bone structure parameters were noted between the sham and OA groups (Figure 11(a)). The OA group had significantly increased BV/TV and Tb.Th and decreased Tb.Sp and Tb.N (Figures 11(b)–11(e)). Treatment with ADSCs or metformin-preconditioned ADSCs prominently alleviated subchondral bone loss. The average value of BV/TV was 0.22 ± 0.01 and 0.23 ± 0.01 in ADSC and metformin-preconditioned ADSC treatment groups, respectively, which were higher than the values in the OA group (0.17 ± 0.02) (*p* < 0.05) at 12 weeks (Figure 11(b)). Tb.N in the ADSC and metformin-preconditioned ADSC groups was higher than that in the OA group (*p* < 0.05) (Figure 11(c)). Additionally, Tb.Sp decreased in the ADSC and metformin-preconditioned ADSC groups (*p* < 0.01) (Figure 11(d)). Furthermore, the value of Tb.Th in the treatment groups did not significantly differ from that in the OA group (Figure 11(e)).

#### 3.6.4. Pain Sensitization

DMM surgery resulted in irregular walking patterns, with a significant decrease in RH/LH print area (Figure 12(a)), max contact area (Figure 12(b)), max contact max intensity (Figure 12(c)), and duty cycle (Figure 12(d)). The max contact max intensity and duty cycle were reduced by the intra-articular injection of ADSCs or metformin-preconditioned ADSCs (Figures 12(c) and 12(d)). These data suggested that the intra-articular injection of ADSCs (preconditioned with metformin or not) partially ameliorates DMM-induced OA pain. The ADSC treatment group and the metformin-preconditioned ADSC treatment group did not significantly differ in these parameters.

## 4. Discussion

In this study, we developed a novel strategy based on a well-known antihyperglycemic agent (metformin) to ameliorate the senescence of ADSCs and then evaluated the efficacy of transplantation with metformin-preconditioned ADSCs to counteract synovial inflammation and prevent articular cartilage lesions in a DMM-induced mouse OA model. Low-dose metformin ameliorated H_2_O_2_-induced senescence of ADSCs by stimulating autophagy via activation of the AMPK/mTOR pathway. Furthermore, mice transplanted with preconditioned cells showed persistent synovial reactivity and reduced cartilage alterations and pain at the endpoint evaluation.

Under oxidative stress or long-term passaging, stem cells undergo senescence with loss of stemness and dysfunction. Metformin not only achieves glycemic control but also exhibits other beneficial effects in cell and organism aging. In our study, we found that low-concentration metformin efficiently prevents the senescence of ADSCs under oxidative stress.

Metformin has been shown to ameliorate the senescence of bone marrow mesenchymal stem cells [23, 24], human diploid fibroblasts [24], lens epithelial cells [25], and nucleus pulposus cells [26]. Consistent with these findings, our results first showed that metformin could slow the aging of murine ADSCs. Cellular senescence is closely related to autophagy. Autophagy plays cytoprotective roles through the turnover of long-lived proteins and scavenging damaged cellular components. Enhanced autophagy may ameliorate cellular senescence [10]. In our study, the levels of autophagy-associated proteins in senescent murine ADSCs were decreased. In contrast, pretreatment of ADSCs with metformin enhanced their autophagy and consequently reduced their senescence despite their subsequent exposure to H_2_O_2_.

Although autophagy is influenced by many different signaling pathways, mTOR and AMPK pathways are two core regulators [27]. mTOR assembles into two complexes, mTORC1 and mTORC2 [28]. mTORC1 is the main autophagy suppressor, while AMPK acts as an activator during the regulation of autophagic activity [29]. mTORC1 kinase inhibits autophagy through both ATG13 and ULK1, which play important roles in autophagosome formation [30].

AMPK activates autophagy by negatively regulating mTORC1 by activating TSC2 and directly inhibiting the phosphorylation of RAPTOR (regulatory-associated protein of mTOR) Ser722 and Ser792 residues [27]. Metformin has been reported to induce autophagy mainly through the AMPK-dependent pathway in various mammalian cells. We found that metformin could simultaneously increase AMPK expression and decrease mTOR expression. Under the influence of the AMPK antagonist compound C, levels of phosphorylated AMPK and autophagy-related proteins were reduced, while the expression level of phosphorylated mTOR increased. These results led us to suggest that metformin protects ADSCs against H_2_O_2_-induced cellular senescence by activating autophagy through the AMPK/mTOR pathway.

Metformin is also reported to activate autophagy through other pathways, such as STAT and SIRT1 signaling pathways [31, 32]. Therefore, it is necessary to conduct further studies on the regulation mechanism of senescence through autophagy induced by metformin.

Senescence is not only accompanied by a decrease in autophagy but also by the excessive production of intracellular ROS [33, 34] and DNA damage [35]. Our data indicated that metformin could reduce the senescence-induced elevation of ROS and protect cells against DNA damage [36, 37]. However, further study is necessary to investigate the underlying relationship and mechanism among aging, autophagy, ROS, and DNA damage.

Cartilage degeneration and synovial inflammation are considered to be key drivers of OA pathophysiology [38]. Based on their paracrine effect, ADSCs have been the focus of an emerging therapeutic agent in cell-based therapy for OA [5]. Although many intra-articular transplantations of ADSCs have demonstrated encouraging outcomes, the senescence of ADSCs should be addressed before or after injection. We found that metformin-preconditioned ADSCs better ameliorated cartilage degeneration and synovial inflammation than ADSCs as, respectively, evident by the lower percentages of chondrocytes positive for MMP-13 and modulation of less synovial macrophage polarization to the M1 phenotype.

Although we did not investigate the underlying mechanism, previous studies have shown that ADSCs express many immune modulators, including interleukin-1 receptor antagonist, interleukin-10, indoleamine 2,3-dioxygenase (IDO), and transforming growth factor-beta, by which they could switch monocytes/macrophages from proinflammatory to anti-inflammatory phenotypes [39]. The precise mechanisms, especially the interaction between ADSCs and chondrocytes or macrophages, deserve further investigation.

ADSCs have always been held in high regard for the treatment of OA, but their effect is limited. Various techniques have been extensively investigated, especially based on immune regulation. In addition to its antidiabetic effect, recent studies have shown that metformin has anti-inflammatory properties. Metformin regulates the immunoregulatory properties of Ad-hMSCs by increasing the expression of IDO and IL-10. However, we found the concentration of metformin used in our study (100 *μ*M) to be much lower than that used in the study of Park et al. (1 mM) [40]. This low-dose metformin treatment was also reported in a recent study [41]. We hypothesized that the dual anti-inflammatory effects of ADSCs and metformin might improve OA treatment by regulating synovial inflammation. Therefore, we proposed a novel strategy of preconditioning ADSCs with metformin before injection for OA treatment.

ADSCs were shown to play an important role in maintaining chondrocyte homeostasis. Stem cells, especially ADSCs, can promote cartilage repair and even regeneration; therefore, they can be used in the treatment of OA [5, 7, 42–45]. Our results were consistent with previous reports. After the intra-articular injection of metformin-preconditioned or not preconditioned ADSCs, OARSI scores in the joints improved. The expression level of chondrogenesis markers collagen II was also upregulated, while the expression level of catabolism markers MMP-13 was reduced. Cartilage degeneration is related to arthritis, and it is considered that the combined functions of the cartilage and subchondral bone affect OA progression. Our micro-CT analysis revealed that metformin-preconditioned or not preconditioned ADSCs attenuated subchondral bone remodeling, but there was no significant difference between ADSCs and metformin-preconditioned ADSCs. Apart from these, pain relief is also critical in the treatment of OA. DMM-induced OA in mice leads to moderate joint biomechanical imbalance. The disease progression is very similar to the clinical manifestations in humans [20]. The main disadvantage of DMM-induced OA is that it requires surgical operation. In addition, due to the small size of the mouse knee joint, the operation process is relatively difficult and requires careful operation, and there is a possibility of postoperative infection. However, considering the animal type, cost, modeling time, length of experiment, and clinical relevance, the mouse model of DMM-induced OA is still a good choice. Thus, the DMM model is an ideal model to evaluate therapeutic effects on OA pain. Gait analysis is a useful tool to understand behavioral changes in preclinical arthritis models [46]. Our findings suggest that pain symptoms can be improved by ADSC therapy.

The need to obtain repeatable results is vital for stem cell-based cytotherapy. There is no doubt that clinical trials of induced pluripotent stem cells are on the forefront [47, 48]. However, derivation, quality attributes, tumorigenicity, and immune rejection of these stem cells are the common challenges [49], similar to stem cells from other sources. Invasive surgery, purification *in vitro*, and specific differentiation condition are the main barriers for ADSCs to be widely used. Apart from this, the *in vivo* fate of transplanted cells is critical for the therapeutic outcome. DiR-labeled ADSCs were evaluated by using a biofluorescence imaging system. The fluorescence could be observed even 7 days after injection. Li et al. [50] reported that DiR-labeled ADSCs persisted for 10 weeks in the rat OA model. These results indicated that the injected cells could survive and be functionally active in the knee joint.

Taken together, our study reveals that metformin preconditioning is an effective and vital approach to optimize ADSC transplantation for OA and provides limited functional benefit for motor function as well.

Although ADSCs have demonstrated good treatment outcomes, many challenges still need to be addressed, including the starting time of intra-articular injection, the frequency of injection, and the number of cells injected each time. In addition, the current treatment strategy only delays disease progression; therefore, cartilage repair and prevention of joint degeneration both need to be achieved using better biomaterials in the future and optimization of experimental conditions.

## 5. Conclusion

Metformin could ameliorate the H_2_O_2_-induced senescence of ADSCs. Our results revealed the mechanisms by which metformin modulates senescence and autophagy in ADSCs. Moreover, metformin-preconditioned ADSCs protected OA mice, thereby showing its therapeutic potential for OA.

## Figures and Tables

**Figure 1:** Characterization of adipose-derived stem cells (ADSCs). (a) ADSCs exhibited a representative spindle-shaped morphology. (b) Representative images showed pluripotent differentiation abilities (osteogenic, adipogenic, and chondrogenic) of ADSCs. Scale bar = 100 *μ*m. (c) Flow cytometry analysis of surface markers on mouse ADSCs. CD29, CD90, and CD105 stained positive, while CD34 and CD45 stained negative.

**Figure 2:** Effects of metformin (100 *μ*M–5 mM) on the viability of ADSCs. Cell viability was determined by the CCK-8 assay. Data represent the mean ± SD (*n* = 4). Using one-way ANOVA, statistically significant differences are indicated by ^∗^*p* < 0.05 and ^∗∗∗^*p* < 0.001.

**Figure 3:** Metformin attenuated H_2_O_2_-induced ADSC senescence. (a) ADSCs were treated with H_2_O_2_ (50–400 *μ*M) for 2 h, and cell viability was measured by the CCK-8 assay. The results are presented as mean ± SD (*n* = 4). Using one-way ANOVA, ^∗∗^*p* < 0.01 and ^∗∗∗^*p* < 0.001 vs. control group. (b) ADSCs were pretreated with metformin at the indicated concentrations for 24 h and then incubated with or without 200 *μ*M H_2_O_2_ for further 2 h. Cell viability was measured by the CCK-8 assay. The results are presented as mean ± SD (*n* = 4). Using one-way ANOVA, ^∗∗^*p* < 0.01 and ^∗∗∗^*p* < 0.001 vs. H_2_O_2_ group. (c) Micrographs of representative cellular senescence were analyzed by SA-*β*-Gal staining, and the quantitation is shown on the right (scale bar = 200 *μ*m). The results are presented as mean ± SD (*n* = 3). Using one-way ANOVA, ^∗∗∗^*p* < 0.001. (d) Protein expression of p21 and p16 was assessed by western blotting (left) and quantitation (right). Data are presented as mean ± SD of at least three separate experiments. Using one-way ANOVA, ^∗∗^*p* < 0.01 vs. control group, ^#^*p* < 0.05 vs. H_2_O_2_ group, and ^&^*p* < 0.05 and ^&&^*p* < 0.01 vs. “MET+H_2_O_2_” group.

**Figure 4:** Metformin alleviates H_2_O_2_-induced ROS generation and DNA damage in ADSCs. (a) The cellular ROS was detected by the probe DCFH-DA under a fluorescence microscope. Scale bar = 100 *μ*m. (b) Representative analysis of ROS levels in ADSCs by flow cytometry (left). The levels of intracellular ROS in ADSCs detected by the DCF-MFI (right). The results are presented as mean ± SD (*n* = 3). Using one-way ANOVA, ^∗∗∗^*p* < 0.001 vs. control group and ^#^*p* < 0.05 and ^##^*p* < 0.01 vs. H_2_O_2_ group. (c) Representative immunofluorescence staining for *γ*H2A.X. Scale bar = 20 *μ*m. (d) Representative western blots show protein levels of Rad51 and *γ*H2A.X. The results are presented as mean ± SD (*n* = 3). Using one-way ANOVA, ^∗∗^*p* < 0.01 and ^∗∗∗^*p* < 0.001 vs. control group and ^#^*p* < 0.05 vs. H_2_O_2_ group.

**Figure 5:** Metformin attenuated H_2_O_2_-induced senescence of ADSCs by activating autophagy. (a) Autophagic corpuscle was detected by transmission electron microscopy. Red arrows indicate the formation of autophagic vacuoles. Scale bar = 2000 nm. (b) ADSCs were treated with different concentrations of metformin for 24 h, and the protein expression of Beclin-1 and LC3B-II/LC3B-I was assessed by western blotting (left) and quantitation (right). (c) The level of autophagy-related protein Beclin-1 and LC3B-II/LC3B-I was assessed by western blot (left) and quantitation (right). Data are presented as mean ± SD of at least three separate experiments. Using one-way ANOVA, ^∗^*p* < 0.05, ^∗∗^*p* < 0.01, and ^∗∗∗^*p* < 0.001 vs. control group, ^#^*p* < 0.05 vs. H_2_O_2_ group, and ^&^*p* < 0.05 and ^&&^*p* < 0.01 vs. “MET+H_2_O_2_” group.

**Figure 6:** Metformin induced autophagy via the AMPK/mTOR pathway. (a) ADSCs were treated with different concentrations of metformin for 24 h, and the protein expression of AMPK, p-AMPK, mTOR, and p-mTOR was assessed by western blotting (left) and quantitation (right). (b) Protein expression of AMPK, p-AMPK, mTOR, and p-mTOR was assessed by western blotting (left) and quantitation (right). Data are presented as mean ± SD of at least three separate experiments. Using one-way ANOVA, ^∗^*p* < 0.05, ^∗∗^*p* < 0.01, and ^∗∗∗^*p* < 0.001 vs. control group, ^##^*p* < 0.01 vs. H_2_O_2_ group, and ^&^*p* < 0.05 vs. “MET+H_2_O_2_” group.

**Figure 7:** (a) In vivo imaging of DiR-labeled ADSCs at 1, 3, and 7 days postinjection. After injection of 2 × 10^4^ DiR-labeled ADSCs, representative images are shown. (b) Quantitation of DiR-labeled ADSC fluorescence signal.

**Figure 8:** Effect of metformin-pretreated ADSCs on cartilage degradation at 12 weeks after DMM surgery. Intra-articular injection of ADSCs was performed biweekly, starting 4 weeks after DMM surgery. (a) The knee joint was harvested at 12 weeks after DMM surgery and analyzed histologically using Safranin O-fast green staining. Scale bar = 200 *μ*m. (b and c) The joint lesions were graded on a scale of 0–6 using the OARSI scoring system. All data are shown as mean ± SD (*n* = 8 − 10). Using one-way ANOVA, ^∗∗∗^*p* < 0.001 vs. sham group, ^#^*p* < 0.05, ^##^*p* < 0.01, and ^###^*p* < 0.001 vs. OA group, and ^&^*p* < 0.05 vs. ADSC group.

**Figure 9:** Metformin partially promoted the therapeutic effect of ADSCs. (a and b) Immunohistochemistry and quantitative analysis of collagen II and MMP-13 in knee sections. Scale bar = 200 *μ*m. All data are shown as mean ± SD (*n* = 8 − 10). Using one-way ANOVA, ^∗∗∗^*p* < 0.001 vs. sham group, ^##^*p* < 0.01 and ^###^*p* < 0.001 vs. OA group, and ^&^*p* < 0.05 vs. ADSC group.

**Figure 10:** Metformin-pretreated ADSCs reduced synovial inflammation. (a) Representative image of H&E staining in the synovial tissue and quantification of synovitis scores. (b–d) Immunohistochemistry and quantification analysis of F4/80, iNOS, and CD206, respectively, in the synovial tissue. Scale bar = 50 *μ*m. Synovial macrophages were identified by F4/80 immunohistochemistry; moreover, iNOS was chosen for marking M1-type macrophages and CD206 for M2-type macrophages. Quantification of the ratio of positive stained synovial macrophages, M1 macrophages, and M2 macrophages, respectively, in synovial tissue. All data are shown as mean ± SD (*n* = 8 − 10). Using one-way ANOVA, ^∗∗∗^*p* < 0.001 vs. sham group, ^#^*p* < 0.05, ^##^*p* < 0.01, and ^###^*p* < 0.001 vs. OA group, and ^&^*p* < 0.05 vs. ADSC group.

**Figure 11:** Evaluation of subchondral change by micro computed tomography. (a) Three-dimensional reconstruction image of tibial subchondral bone in each experimental group at 12 weeks after Sham or DMM operation. (b) Quantitative analysis of bone volume/tissue volume (BV/TV). (c) Quantitative analysis of trabecular number (Tb.N). (d) Quantitative analysis of trabecular separation (Tb.Sp). (e) Quantitative analysis of trabecular thickness (Tb.Th). All data are shown as mean ± SD (*n* = 3). Using one-way ANOVA, ^∗^*p* < 0.05 and ^∗∗∗^*p* < 0.001 compared with the sham group and ^#^*p* < 0.05 and ^##^*p* < 0.01 compared with the OA group.

**Figure 12:** Functional assessment by catwalk analysis. (a) Paw print area, (b) max contact area, (c) max contact max intensity, (d) duty cycle, (e) mean intensity, (f) stand, and (g) swing speed were analyzed at 12 weeks after sham or DMM operation. Data are expressed as mean ± SD (*n* = 8). Using one-way ANOVA, ^∗^*p* < 0.05 vs. sham group and ^#^*p* < 0.05 vs. OA group.

## Data Availability

Data generated from this work and presented in this manuscript is available upon request from the corresponding author.
